The article "Importance of Follow-Up Cerebrospinal Fluid Analysis in Cryptococcal Meningoencephalitis" was published in 2014. Journal: Dis Markers.

# Importance of Follow-Up Cerebrospinal Fluid Analysis in Cryptococcal Meningoencephalitis

**DOI:** 10.1155/2014/162576

**Published:** 2014-10-13

**Authors:** Thomas Skripuletz, Philipp Schwenkenbecher, Kaweh Pars, Matthias Stoll, Josef Conzen, Seza Bolat, Refik Pul, Ralf-Peter Vonberg, Ludwig Sedlacek, Ulrich Wurster, Martin Stangel, Corinna Trebst

**Affiliations:** ^1^Department of Neurology, Hannover Medical School, Carl-Neuberg-Straße-1, 30625 Hanover, Germany; ^2^Department of Immunology and Rheumatology, Hannover Medical School, 30625 Hannover, Germany; ^3^Department of Diagnostic and Interventional Neuroradiology, Hannover Medical School, 30625 Hannover, Germany; ^4^Department of Neurology, University of Lübeck, 23538 Lübeck, Germany; ^5^Institute for Medical Microbiology and Hospital Epidemiology, Hannover Medical School, 30625 Hannover, Germany

## Abstract

Cryptococcal meningoencephalitis represents a serious infection of the central nervous system, where reliable prognostic factors during the disease course are needed. Twenty-one patients diagnosed with cryptococcal meningoencephalitis in a German university hospital from 1999 to 2013 were analysed retrospectively. CSF parameters were analysed prior to therapy and during antifungal treatment and were compared between patients who survived or deceased. Fifteen patients clinically improved after antifungal therapy, while six patients died. No differences were observed between the outcome groups for the CSF parameters cell count, lactate, total protein, and CSF-serum albumin quotients (QAlb). Follow-up examinations of serum cryptococcal antigen titer and CSF cell count have shown that these parameters cannot be used to monitor the efficacy of antifungal therapy as well. In contrast, the course of QAlb during therapy was indicative for the outcome as a possible prognostic marker. In patients with clinical improvement QAlb values were falling under therapy, while rising QAlb values were found in patients with fatal outcome indicating a continuing dysfunction of the blood-CSF barrier. In conclusion, our results indicate that, among the various CSF parameters, the course of QAlb presents a promising marker that might be used to monitor the efficacy of antifungal therapy.

## 1. Introduction

Cryptococcal meningoencephalitis presents a serious life-threatening infection of the central nervous system (CNS) in patients with both intact and compromised immune system [1]. It is a common opportunistic infection and AIDS-defining illness in patients with HIV infection. Before the highly active antiretroviral therapy (HAART) era, the prevalence of AIDS associated cryptococcal meningoencephalitis was 5–10% in the developed countries [2, 3]. Following the introduction of combination antiretroviral therapy, the incidence of cryptococcosis has declined substantially [4]. However, despite antiretroviral treatment and appropriate antifungal therapy, the mortality remains high even in the developed countries ranging from 10 to 30% [5–7]. Thus, further strategies for improving the overall outcome are needed.

The article "Importance of Follow-Up Cerebrospinal Fluid Analysis in Cryptococcal Meningoencephalitis" was published in 2014. Journal: Dis Markers.

In addition, there is a need for reliable prognostic factors during the disease course. Several baseline characteristics such as severity of illness, immunological status, and renal and liver function were thought to influence the prognosis but a clear association with the clinical outcome could not be found [8, 9]. Since clinical data at admission appear unreliable as prognostic marker, analysis of the cerebrospinal fluid (CSF) might present another interesting tool. CSF examination is generally considered a key procedure in the diagnosis of CNS infections [10]. Results of CSF analyses, in particular CSF cell counts, glucose, lactate, and total protein levels, were previously reported in various series of patients with cryptococcal meningoencephalitis [11]. However, no study has, to date, specifically evaluated a potential relationship of the CSF parameters during disease course with the clinical outcome. Furthermore, several advanced CSF parameters, such as CSF-serum albumin quotient and intrathecal synthesis of the immunoglobulins IgG, IgA, and IgM, were not evaluated in series of patients with cryptococcal meningoencephalitis in contrast to other CNS infections where the beneficial contribution of the CSF has been clearly established [12].

Here, we performed a thorough evaluation of the cerebrospinal fluid data in patients with cryptococcal meningoencephalitis. In addition to baseline values prior to antifungal therapy, follow-up analyses during the disease course were included.

## 2. Materials and Methods

### 2.1. Patients

The retrospectively evaluated data originate from twenty-one patients collected for routine diagnosis in the Hannover Medical School in the time from 1999 to 2013. Eighteen patients were of Caucasian origin, while two patients were born in Thailand and migrated to Germany three or eleven years before, and one patient was born in Kenya and migrated to Germany fourteen years before. One patient was not included in the study due to insufficient clinical and laboratory data. One patient included in the present study was described in detail before [13]. Cryptococcal meningitis was defined as either positive CSF cryptococcal antigen titer or cultural growth of cryptococcus from CSF. Results from the initial CSF analysis were available from all patients. During follow-up twenty-eight further CSF examinations were available from thirteen patients.

The article "Importance of Follow-Up Cerebrospinal Fluid Analysis in Cryptococcal Meningoencephalitis" was published in 2014. Journal: Dis Markers.

The investigation was approved by the local ethics committee of the Hannover Medical School. This is a retrospective study and only data were included that were evaluated for patients treatment.

### 2.2. CSF Analytical Procedures

CSF and serum were analysed by standard methods. CSF cell count, total protein, and lactate were analysed immediately after CSF withdrawal by lumbar puncture. CSF leukocytes were counted manually with a Fuchs-Rosenthal counting chamber. A white cell count ≥5 cells/*μ*L was considered elevated. For further analyses the residual CSF was centrifuged (145 g for 15 min) and the supernatant frozen at −70°C. Total protein was determined by the Bradford dye-binding procedure. The method involves the binding of Coomassie Brilliant Blue G-250 to proteins (primarily to basic and aromatic amino acid residues) producing a colour change. Optical density was measured with a spectrophotometer (Beckman Coulter DU730) and then compared to a standard curve of known protein concentrations. Albumin, IgG, IgA, and IgM in CSF and serum were determined together in the same latex enhanced assay by kinetic nephelometry on a Beckman Coulter IMMAGE Immunochemistry System. Albumin quotients (QAlb) were calculated using the formula CSF albumin/serum albumin (QAlb = CSF albumin/serum albumin) in order to assess the blood-CSF barrier function. The age-adjusted upper reference limit of QAlb was calculated using the formula QAlb = 4 + (age in years/15) [14]. Intrathecal synthesis of IgG, IgA, and IgM was calculated based on the method of Reiber-Felgenhauer referring the IgG, IgA, and IgM CSF/serum quotients to the albumin quotient [14]. CSF-specific oligoclonal bands (OCB) were determined by isoelectric focusing in polyacrylamide gels with consecutive silver staining. For all protein analyses, CSF and serum samples were analysed within the same analytical series. All methods are quality assured by participating in external quality control programs, the CSF survey of INSTAND [15].

### 2.3. Cerebral Magnetic Resonance Imaging

All patients were examined by cerebral magnetic resonance imaging (MRI) at baseline. In addition to the standard screening procedures, the images were inspected for typical cryptococcal related lesions: dilatated Virchow-Robin spaces, pseudocysts, parenchymal nodules/cryptococcomas, hydrocephalus, and radiological signs of vasculitis and meningitis [16]. All measurements included a T1-weighted sequence and an axial fluid-attenuated inversion recovery (FLAIR). A T2-weighted sequence was performed either sagittally or axially. Contrast medium was applied in all except for two patients due to incompliance. During the disease course thirty-nine further radiological examinations of the brain were performed in thirteen patients (eight survivors and five nonsurvivors). Ten patients were scanned by MRI of whom five received additional CT scans and three patients were analysed by CT scans of the brain only.

The article "Importance of Follow-Up Cerebrospinal Fluid Analysis in Cryptococcal Meningoencephalitis" was published in 2014. Journal: Dis Markers.

### 2.4. Statistical Analysis

GraphPad Prism version 5.02 was used for statistical analysis. Adobe Illustrator CS4 14.0 was used to arrange figures. For comparison of two independent groups, the two-tailed unpaired two-sided Mann-Whitney test was performed. In order to predict the course of cerebrospinal fluid parameters, simple linear regression was performed and slopes were analysed whether they are significantly different from zero. For each comparison, a *P* value < 0.05 was considered as statistically significant.

## 3. Results

### 3.1. Patients Characteristics

In the period from 1999 to 2013, twenty-one patients were diagnosed with cryptococcal CNS infection. The male gender was predominant and only five females were identified (Table 1). Our patients were categorized into two groups according to the outcome with regard to mortality (Table 1).

Seventeen patients suffered from HIV infection as a predisposing factor for cryptococcal meningitis. Of those patients, seven had been diagnosed with HIV before the presentation of cryptococcal meningitis, but only two patients were treated with antiretroviral therapy (ART) at admission. Four patients with known HIV infection had a previous AIDS-defining illness (Table 2). The majority of HIV-infected patients (65%) presented with concurrent infections at admission (Table 2). All but two patients in the HIV-infected group had a viral load >30,000 copies/mL in serum. In all but two patients, the CD4 counts were <50/mm^3^.

In the HIV negative group three patients had risk factors such as kidney transplant with immunosuppressive treatment nine months previously, idiopathic lymphocytopenia and chronic polyarthritis with use of corticosteroids for one year, and autoimmune hemolytic anemia with use of corticosteroids for eighteen years.

### 3.2. Neurologic Signs and Symptoms

All patients had at least one symptom at minimum that led to a diagnostic lumbar puncture. Headache (71%), disturbance of consciousness (62%), fever (48%), and nausea with vomiting (38%) were found as the most common symptoms at admission (Table 1). All patients suffered from either disturbance of consciousness or headache but the combination of both was found only in 33% of patients. Stiff neck as a typical sign of meningitis was quite rare and occurred only in three patients. Focal neurologic deficits such as aphasia and ataxia were also rare and found in three patients. One patient presented with an epileptic seizure.

The article "Importance of Follow-Up Cerebrospinal Fluid Analysis in Cryptococcal Meningoencephalitis" was published in 2014. Journal: Dis Markers.

### 3.3. Complications during the Course of Treatment

All patients were treated with liposomal amphotericin B (1–4 mg/kg i.v. OD) + flucytosine (25 mg/kg i.v. QID), while all but one were additionally treated with fluconazole (200–400 mg i.v./p.o. BID) as recommended by local guidelines [17]. In patients with clinical improvement antifungal treatment was performed over a time period of 4-5 weeks in seven patients, 5-6 weeks in two patients, and 6–10 weeks in six patients.

The mortality rate was high in our cohort as six patients died (29%; four of them were infected with HIV). The six patients with treatment failure died within 3, 4, 5, 6, 11, or 14 weeks of therapy with a triple combination of liposomal amphotericin B + flucytosine + fluconazole. All six patients developed a progressive disturbance of consciousness before death. Two of them suffered multiple cerebral infarctions and two patients had epileptic seizures with increasing frequency.

In patients that survived, neurological complications were found rarely during therapy. One patient developed new seizures and one other patient presented with abducens nerve palsy. Frequent nonneurologic complications during disease course in these patients included electrolyte disturbance (100%), elevated transaminases (81%), hypercreatinemia (52%), and allergic reactions (10%).

### 3.4. Neuroimaging Findings

Pseudocysts as typical signs of cryptococcal CNS infection [16, 18] were found in six patients, while dilatated Virchow-Robin spaces were found in four patients (Figure 1 and Table 3). Pseudocysts were localized predominantly in the basal ganglia and rarely paraventricular and supraventricular. Parenchymal nodules/cryptococcomas as another typical sign of cryptococcal CNS infection [16, 18] were not identified in our patients. Radiological signs of meningitis as defined by meningeal contrast enhancement were rare and found only in three patients of whom one had a fatal outcome. Signs of basal vasculitis were found in two patients with fatal outcome; in both of these patients multiple cerebral infarctions localized in the basal ganglia and mesencephalon were identified. One patient with good outcome showed a lacunar infarction of the right nucleus caudatus but no signs of basal vasculitis. Hydrocephalus which might occur as complication of cryptococcal CNS infection was found in three patients of whom one did not survive (this patient had a basal vasculitis and multiple infarctions). Signs of HIV-encephalopathy were found in only one patient while seven patients presented with cerebral atrophy.

The article "Importance of Follow-Up Cerebrospinal Fluid Analysis in Cryptococcal Meningoencephalitis" was published in 2014. Journal: Dis Markers.

During disease course only one patient with clinical improvement showed a new MRI finding (signs of meningitis). In contrast, two patients with fatal outcome showed progressive cerebral infarctions. Both patients had no infarctions at baseline MRI. One other patient with fatal outcome showed pseudocysts and signs of meningitis.

### 3.5. Cerebrospinal Fluid Analyses

Eighteen patients (86%) were identified with increased cell counts (Table 4). Thirteen patients (62%) presented low increased cell numbers between 5 and 200/*μ*L, while five (24%) showed cell counts between 200 and 900/*μ*L. In three patients normal cell counts with 1–3 cells/*μ*L were found; all patients were infected with HIV.

Lactate concentration in the CSF was normal in only two patients infected with HIV. All other cases had an elevated CSF lactate concentration (>2.6 mmol/L).

Total CSF protein was found within the normal range of 200–500 mg/L in only three patients. Ten patients (48%) presented CSF protein levels that were mildly increased within a range of 500–1000 mg/L, while eight patients (38%) showed values >1000 mg/L.

Since measurement of total protein levels in the CSF may show normal results despite a blood-CSF barrier dysfunction [19], the albumin CSF-serum concentration quotient (QAlb) was analysed. QAlb is generally accepted as the best indicator to describe a blood-CSF barrier dysfunction for blood derived proteins [14]. QAlb values within the normal range were found in three patients. In eighteen patients (86%) there was an elevated QAlb indicating a blood-CSF barrier dysfunction. Barrier dysfunction was severe in six patients (QAlb > 20) and mild to moderate in the other patients.

For the cerebrospinal fluid parameters cell count, lactate, total protein, and QAlb, no significant differences between the outcome groups were found indicating that baseline CSF analysis prior to antifungal therapy is not helpful as prognostic marker.

Intrathecal immunoglobulin (Ig) synthesis of IgG as calculated based on the method of Reiber-Felgenhauer [14] was observed in four patients. One patient was identified in the survivor group (7%), while three patients were found in the group with fatal outcome (50%). Intrathecal IgA synthesis was found in one patient with treatment failure (17%). Intrathecal IgM synthesis was found in five patients, two with clinical improvement (13%), and three with fatal outcome (50%).

CSF-specific oligoclonal bands were determined by isoelectric focusing, which is the most sensitive method to detect intrathecal IgG synthesis in the CSF. Twelve patients (57%) showed oligoclonal bands restricted to the CSF. Eight patients were identified in the survivor group (53%), while four patients were found in the group with fatal outcome (67%).

The article "Importance of Follow-Up Cerebrospinal Fluid Analysis in Cryptococcal Meningoencephalitis" was published in 2014. Journal: Dis Markers.

Identical oligoclonal IgG bands in CSF and serum were found in eleven patients (52%). From these eleven patients nine survived (88%). Six of these eleven patients showed a combination of oligoclonal bands restricted to the CSF and oligoclonal IgG bands in CSF and serum. Identical oligoclonal IgG bands are the result of a systemic humoral immune response towards foreign antigens and/or self-antigens. Identical oligoclonal IgG bands are commonly found in subacute systemic infections and confirm the presence of a strong immune reaction in patients with cryptococcal infection.

In four patients (19%) no oligoclonal bands in either the CSF or serum were found.

### 3.6. Course of Cryptococcal Antigen Titers

Before treatment and during disease course cryptococcal antigen titers were analysed predominantly in the serum and fifty-eight values from sixteen patients (ten survived patients and six patients with outcome death) were available. The cryptococcal antigen latex agglutination tests were positive before therapy with titers ranging from 1 : 2 to 1 : 65536. During disease course cryptococcal antigen titers decreased up to 3 log steps in eight patients or were stable in four patients. A decrease occurred even in two patients with failed therapy. An increase in cryptococcal antigen titers up to 3 log steps occurred in three patients with clinical improvement while one patient with fatal outcome presented with increased titers of 6 log steps. Thus, these results indicate that the antigen titer cannot be used to monitor the efficacy of antifungal therapy with regard to mortality.

### 3.7. Course of CSF-Serum Albumin Quotient as a Possible Prognostic Marker for Mortality

During antifungal therapy cell counts decreased in all patients that had an increased cell count before (three patients had a normal cell count of 1–3/*μ*L before therapy). The decrease occurred even in patients with failed therapy indicating that cell count is not a useful value to monitor the efficacy of antifungal therapy with regard to mortality (Figure 2(a)).

Measurements of total protein levels in the CSF during disease course showed decreasing values in the majority of patients with clinical improvement, while two patients had a stable value and one patient had a small increase (Figure 2(b), slope of regression curve not significant). In contrast, patients with the outcome death presented increasing total protein values (slope of regression curve differs from zero significantly *P* = 0.02).

Analysis of QAlb revealed decreasing values in all patients with clinical improvement (Figure 2(c), slope of regression curve not significant), while increasing QAlb values were found in all patients with fatal outcome (Figure 2(c), slope of regression curve differs significantly from zero *P* = 0.04). Thus, in our cohort the course of QAlb values arises for a possible prognostic marker for the clinical outcome.

The article "Importance of Follow-Up Cerebrospinal Fluid Analysis in Cryptococcal Meningoencephalitis" was published in 2014. Journal: Dis Markers.

During follow-up, four patients with a favorable outcome showed a new intrathecal synthesis of immunoglobulins (IgM in two patients; combined IgG and IgA in two patients). In contrast, in two patients with fatal outcome intrathecal synthesis of IgM and IgG disappeared.

During disease course one additional patient developed oligoclonal bands restricted to the CSF and one additional patient showed identical oligoclonal IgG bands detected in CSF and serum. Both patients showed a clinical improvement.

## 4. Discussion

Here, we analysed retrospectively characteristics of clinical presentation, MRI examination of the brain, and cerebrospinal fluid analysis in patients with cryptococcal meningoencephalitis in a German university hospital from 1999 to 2013. Based on the outcome of this population we identified the course of QAlb (either rise or decrease, resp.) in follow-up examinations as a possible prognostic marker.

In our cohort, symptoms on presentation included mostly headache and disturbance of consciousness followed by fever and nausea with vomiting. Stiff neck as a typical sign of meningitis was rare and occurred only in three patients. Focal neurologic deficits were also rare and were only found in three patients. However, during the disease course and antifungal treatment additional symptoms occurred that were predominantly found in patients with fatal outcome. The deceased patients developed a progressive consciousness disturbance before death. Two patients developed progressive cerebral infarctions and two patients had epileptic seizures with increasing frequency. The mortality rate of 29% was high, which is similar to other series of patients described [5–7]. In contrast, during disease course patients who survived only rarely developed neurological complications as new seizures and abducens nerve palsy was found in two patients, respectively.

Brain imaging analyses prior to therapy were abnormal in all patients. Typical signs of cryptococcal CNS infection such as pseudocysts were found in both outcome groups. Interestingly, signs of basal vasculitis were found in two patients with fatal outcome only; in both of these patients multiple cerebral infarctions were identified. During follow-up two patients with fatal outcome presented progressive cerebral infarctions while signs of meningitis were found in another patient. In contrast, in patients with good outcome new changes (signs of meningitis) were found in only one patient.

The article "Importance of Follow-Up Cerebrospinal Fluid Analysis in Cryptococcal Meningoencephalitis" was published in 2014. Journal: Dis Markers.

Detection of cryptococcal antigen is highly specific for the diagnosis of cryptococcal infection [20, 21]. However, follow-up measurements of serum cryptococcal antigen titers in our patients have shown that the antigen titer cannot be used to monitor the acute efficacy of antifungal therapy. We found decreasing antigen titers in two patients with fatal outcome during therapy that led to the misleading suggestion of pathogen clearance. On the other side, three patients with clinical improvement had increasing cryptococcal antigen titers during therapy. Our results are in line with previous reports [22–25] and it was thus recommended that follow-up antigen titers are not useful as prognostic marker during therapy.

Regarding cerebrospinal fluid analysis we did not find significant differences for the parameters cell count, lactate, total protein, and QAlb between the outcome groups indicating that baseline CSF values prior to therapy are not helpful as prognostic marker. During antifungal therapy CSF cell counts decreased in all patients even in those with fatal outcome indicating that the course of cell count is not useful to monitor the efficacy of antifungal therapy as well. In contrast, analysis of QAlb revealed decreasing values in all patients with clinical improvement, while increasing QAlb values were found in all patients with fatal outcome. Thus, in respect to the size of our cohort, the course of QAlb values during therapy might present a possible prognostic marker for the clinical outcome. A similar result was observed for the course of CSF total protein during therapy between the outcome groups. However, during therapy three patients with clinical improvement did not show a decrease of CSF total protein. Measurement of total protein levels in the CSF has some disadvantages, although examinations of total protein are simple and quickly available. Analysis of total protein in the CSF may show normal results despite a blood-CSF barrier dysfunction, because it does not take into account the serum protein level [19]. The total protein concentration in the CSF depends on patients serum protein concentration, the age, the CSF flow rate, and the assay type [14]. Severe inflammatory disorders frequently lead to kidney damage and thus to considerable loss of plasma proteins by excretion into the urine. Accordingly, in our cohort, thirteen patients showed decreased baseline levels of serum albumin (18–34 g/L; reference 35–52 g/L) which is the major fraction of serum total protein. Three of these patients presented with CSF total protein levels within the normal range leading to the misleading suggestion of an intact blood-CSF barrier. However, all of them had a blood-CSF barrier dysfunction as shown by an elevated QAlb. Albumin is exclusively produced in the liver and albumin found in the CSF exclusively originates from the blood. QAlb is therefore generally accepted as the best indicator to describe a blood-CSF barrier dysfunction for blood derived proteins [14]. Thus, we recommend incorporation of QAlb analysis in all CSF examinations.

The article "Importance of Follow-Up Cerebrospinal Fluid Analysis in Cryptococcal Meningoencephalitis" was published in 2014. Journal: Dis Markers.

CSF-specific oligoclonal bands were determined by isoelectric focusing in order to qualitatively detect IgG synthesis in the CSF. In our cohort twelve patients (57%) showed oligoclonal bands restricted to the CSF indicating a local IgG synthesis. Both outcome groups showed similar results as CSF oligoclonal bands were found in eight of fifteen patients with clinical improvement and four of six patients with fatal outcome. CSF oligoclonal bands are the result of humoral immune response in the CNS towards foreign antigens and/or self-antigens. Oligoclonal bands are frequently found in chronic inflammatory diseases of the CNS such as multiple sclerosis or neurosyphilis [14, 26] and confirm the presence of a CNS immune reaction in patients with cryptococcal meningoencephalitis.

Intrathecal synthesis of IgA as calculated based on the method of Reiber-Felgenhauer is a typical finding in patients with neurotuberculosis [26], which is an important differential diagnosis. In our patients IgA synthesis was found only in one patient at baseline prior to therapy and in two additional patients during disease course. However, in all three patients intrathecal IgA synthesis did not occur alone and was always combined with IgG synthesis. Intrathecal synthesis of IgM was found in five patients prior to therapy (three patients with good outcome and two patients with outcome death). Interestingly, during disease course two patients with a favorable outcome showed a new intrathecal synthesis of IgM while in two patients with fatal outcome intrathecal synthesis of IgM disappeared. Intrathecal IgM synthesis is frequently found in patients with neuroborreliosis and mumps meningoencephalitis [26]. To date, the role of intrathecal IgM synthesis was not described in patients with cryptococcal meningoencephalitis. However, it can be speculated that the outcome of this severe CNS infection might be associated with the presence of an intrathecal IgM synthesis.

## 5. Conclusions

In view of the small number of twenty-one patients, we realize the limitations of our observation. Nevertheless, the present study shows that cryptococcal meningoencephalitis is associated with prominent CSF abnormalities. Our results indicate that beside careful clinical observation CSF examinations may allow monitoring disease activity during antifungal therapy. Among the various CSF parameters, the course of QAlb values presents a promising marker that can be used to monitor the efficacy of antifungal therapy.

The article "Importance of Follow-Up Cerebrospinal Fluid Analysis in Cryptococcal Meningoencephalitis" was published in 2014. Journal: Dis Markers.

## Figures and Tables

**Figure 1:** Examples of abnormal neuroradiological findings in cryptococcal meningoencephalitis. (a) presents the typical pattern of cryptococcal gelatinous pseudocysts located in lentiform and caudate nuclei (T2WI hyperintense signal) while T1WI sequences ((b), arrow head) show a hypointense signal without enhancement in the T1 C+ image ((c), arrow head). Signs of meningitis are shown by leptomeningeal enhancement in the cerebellar Gyri in axial ((d), arrow heads) and coronal (e) T1 C+ scans. (f) presents signs of basal meningitis demonstrated by leptomeningeal enhancement (arrow head). Hydrocephalus is shown in axial FLAIR sequences in (g) and (h). The enlargement of the frontal and dorsal horns of the lateral ventricles with a hyperintense rim of the periventricular white matter indicates a CSF extravasation. A CCT scan performed 5 days later shows increased ballooning of the third ventricle and a progressive enlargement of the lateral ventricles (i).

**Figure 2:** Illustration of CSF parameters in cryptococcal meningoencephalitis. In (a) values present CSF cell counts while (b)-(c) show values of total CSF protein and CSF-serum albumin quotient (QAlb) after onset of symptoms and during disease course and antifungal therapy. Initial CSF analysis was performed in all patients, while during follow-up CSF was analysed in thirteen patients (eight patients with good outcome and five patients with fatal outcome). Black points mark values of patients with clinical improvement, while red triangles indicate values of patients with the outcome death. On the right side additional graphs present mean values and standard deviation of both groups in the course of antifungal therapy.

**Table 1:** Patient's characteristics.

Parameter	All patients (*n* = 21)	Survivors (*n* = 15)	Nonsurvivors (*n* = 6)
Characteristics			
Age, years (mean)	44 (±16)	43 (±16)	46 (±17)
Male (no.)	16	11	5
Duration of symptoms to diagnosis, days (mean)	16 (±13)	16 (±16)	16 (±6)
Symptoms on presentation			
Headache (no.)	15	12	3
Disturbance of consciousness (no.)	13	9	4
Fever (no.)	10	6	4
Nausea and vomiting (no.)	8	8	0
Focal neurologic deficits (no.)	3	3^a^	0
Stiff neck (no.)	3	2	1
Seizures (no.)	1	0	1
Complications during hospitalization			
Neurologic complications			
Progressive consciousness disturbance (no.)	6	0	6
Seizures (no.)	3	1	2
Focal neurologic deficits (no.)	3	1^b^	2^c^
Cerebral infarction (no.)	2	0	2
Nonneurologic complications			
Electrolyte disturbance (no.)	21	15	6
Elevated transaminases (no.)	17	13	4
Hypercreatinemia (no.)	11	8	3
Allergic reaction (no.)	2	2	0

^a^Focal neurologic deficits: aphasia (3/3) and ataxia (1/3).

^b^Focal neurologic deficit: abducens nerve palsy (1/1).

^c^Focal neurologic deficit: abducens nerve palsy (2/2) and facial palsy (1/2).

The article "Importance of Follow-Up Cerebrospinal Fluid Analysis in Cryptococcal Meningoencephalitis" was published in 2014. Journal: Dis Markers.

Age and duration of symptoms to diagnosis are presented by mean value and standard deviation.

**Table 2:** Characteristics of HIV infected patients.

	All HIV patients (*n* = 17)	Survivors (*n* = 13)	Nonsurvivors (*n* = 4)
Characteristics in the HIV group			
Previous HIV diagnosis (no.)	7	5	2
Previous AIDS-defining illness (no.)	4	3^a^	1^b^
On ART while onset of symptoms (no.)	2	1	1
Concurrent infections on admission (no.)	11	7^c^	4^d^
Laboratory findings on presentation			
Serum HIV viral load (log⁡10 copies/mL)	5.48 (5.50)	5.50 (5.50)	5.40 (5.53)
CD4 count (cells/*µ*L)	43.38 (60.62)	41.75 (61.01)	48.25 (68.44)
T4/T8 ratio	0.08 (0.07)	0.07 (0.07)	0.09 (0.09)

^a^AIDS-defining illness: pneumocystis jiroveci pneumonia (1/3), progressive multifocal encephalopathy (1/3), and wasting syndrome (1/3).

^b^AIDS-defining illness: pneumocystis jiroveci pneumonia (1/1).

^c^Concurrent infections: candidiasis (6/7), cytomegalovirus infection (3/7), cryptosporidiosis (1/7), and hepatitis C (1/7).

^d^Concurrent infections: candidiasis (4/4) and cytomegalovirus infection (1/4).

Laboratory findings are presented by mean value and standard deviation.

**Table 3:** Neuroimaging findings.

Neuroradiological findings	All patients (*n* = 21)	Survivors (*n* = 15)	Nonsurvivors (*n* = 6)
Pseudocysts (no.)	6	4	2
Dilated Virchow-Robin spaces (no.)	4	4	0
Parenchymal nodules/cryptococcomas (no.)	0	0	0
Radiological meningitis (no.)	3	2	1
Basal vasculitis (no.)	2	0	2
Cerebral infarction (no.)	3	1	2
Hydrocephalus (no.)	3	2	1
Hyperintense T2W signals (no.)	12	10	2
HIV-encephalopathy (no.)	1	1	0
Cerebral atrophy (no.)	7	5	2

Neuroradiological analysis of magnetic resonance image scans of the brain collected at baseline from twenty-one patients infected with cryptococcal meningoencephalitis.

**Table 4:** Cerebrospinal fluid.

Parameter	All patients (*n* = 21)	Survivors (*n* = 15)	Nonsurvivors (*n* = 6)
Leukocytes CSF (cells/*µ*L)	151 (±221)	158 (±256)	132 (±103)
Lactate CSF (mmol/L)	3.6 (±1.1)	3.5 (±0.9)	4.0 (±1.6)
Protein CSF (mg/L)	1074 (±734)	1071 (±793)	1081 (±627)
Albumin quotient CSF/serum	18.7 (±15.0)	18.9 (±15.1)	18.3 (±16.3)
IgG synthesis CSF (no.)	4	1	3
IgA synthesis CSF (no.)	1	0	1
IgM synthesis CSF (no.)	5	3	2
CSF oligoclonal bands (no.)	12	8	4

Baseline cerebrospinal fluid (CSF) results from patients infected with cryptococcal meningoencephalitis prior to therapy. Laboratory findings are presented by mean value and standard deviation.
